# Value Analysis of Neoadjuvant Radiotherapy for Breast Cancer after Modified Radical Mastectomy Based on Data Mining

**DOI:** 10.1155/2022/6257536

**Published:** 2022-05-04

**Authors:** Bo Liu, Haiyun Huang, Lijuan Pan, Yufeng Ma

**Affiliations:** ^1^Department of Breast Surgery, Gansu Provincial Hospital, Lanzhou 730000, Gansu, China; ^2^Department of Orthopedics, Gansu Provincial Hospital, Lanzhou 730000, Gansu, China; ^3^Department of Traditional Medicine, Gansu Provincial Hospital, Lanzhou 730000, Gansu, China

## Abstract

Over the last two generations, there has been a surge of interest in nonmutilating treatment for women with early breast cancer. Neoadjuvant radiation therapy, which is progressively being provided to breast cancer patients, could be used to decrease tumor burden while also providing an ability to examine treatment response. This paper aims to explore the effects of the initiation time of radiotherapy after modified adjuvant radical mastectomy on the prognosis of breast cancer. The EMR data can be used to mine hidden rules, which are of great significance for treatment and prognosis analysis. In collaboration with breast cancer, the appropriate prediction model and visualization method are selected and a visual analysis system for breast cancer group and treatment plan based on electronic medical record is constructed. Patients with multiple dimensions are reduced and clustered to form patient groups. The differences of characteristics among patient groups are intuitively displayed by using Nightingale diagram, word cloud, and time axis visualization methods. The support vector machine (SVM) model is used to predict the treatment scheme. The radiotherapy time after modified radical surgery in the two groups was within 15 weeks (observation group) and 15 weeks (routine group), respectively. The incidence of complications, local recurrence rate, progression-free survival, and quality of life scores of patients in the routine group and observation group were compared. The total incidence of complications differed significantly between the observation and routine groups. The physical function, material function, psychological function, and social function of the observation group were significantly higher than the routine group (*P* < 0.05). Radiotherapy within 15 weeks after modified radical mastectomy for breast cancer can not only reduce the local recurrence rate but also prolong the progression-free survival of patients, and the incidence of complications will not increase, which will greatly help improve the quality of life of patients.

## 1. Introduction

Breast cancer is a common disease among women and is the highly prevalent cancer type in the world. Breast cancer is one of the most common malignant tumors that pose a major threat to women's health. The process of metastasis and infiltration of breast cancer is complex and can affect the quality of survival of patients [1]. In many cases, after diagnosis, the patient's disease has already reached a locally advanced stage and the best time for treatment has been missed. Neoadjuvant chemotherapy followed by modified radical surgery and radiotherapy after surgery is needed to prevent distant metastasis and local recurrence [2]. Numerous clinical studies have shown that postoperative radiotherapy can help improve the prognosis of breast cancer patients. However, there are still different opinions on the timing of postoperative radiotherapy [3]. In this paper, we investigated 60 patients admitted to our hospital after modified radical surgery for breast cancer after neoadjuvant chemotherapy, from August 2018 to August 2019, to investigate the best time to start radiotherapy.

With the advancement of medical treatment, breast cancer treatment technology has been developed to a great extent, not only in terms of drug treatment with trastuzumab, an anti-HER2 target [4], but also in terms of surgery, from extended radical breast cancer surgery to less invasive breast-conserving surgery [5]. However, breast cancer is a complex pathological change due to multiple genetic alterations, and the pathological and clinical features vary from patient to patient. In the molecular staging of breast cancer, breast cancer is classified into Luminal A, Luminal B, HER2 overexpressing, and basal-like types according to the estrogen receptor, progesterone receptor, and HER2 expression levels, and different molecular staging has a different prognosis and corresponding therapeutic means [6].

“Precision” diagnosis and treatment are based on “precise” genetic testing and bioinformatics analysis, such as genomics, proteomics, imaging, patronymics, etc., to specifically determine the pathogenesis of tumors. It is also used to select the corresponding surgical methods or targeted therapeutic drugs, achieve “precise” resection of tumors and precise medication for the target, and form patient-centered individualized medical treatment [7].

In 2011, the National Academy of Sciences officially introduced the concept of precision medicine. Since 2016, there has been an explosion in breast cancer-related research worldwide [8].

In the treatment of breast cancer, the traditional methods are to locate and diagnose the suspected lesion through medical history, physical examination, ultrasound, mammography, magnetic resonance imaging, pathology, and other examination methods and then adopt corresponding surgery, chemotherapy, radiotherapy, endocrine therapy, targeted therapy, and other comprehensive treatment methods. With the development of information technology, the rapid analysis of massive data has become a reality. The precision diagnosis and treatment based on medical big data have gradually become the future development trend, especially under the transformation of the current 5P medical model. It has become a fundamental leader in the development of accurate prevention, prediction, and personalized medical services. The root of the realization of this model lies in the integrated processing of medical big data and the development of intelligent algorithms [9]. Among them, the mammography image recognition technology developed based on imaging histology has effectively completed the intelligent diagnosis of a breast cancer diagnosis. It is expected to solve the problem of regional diagnostic level imbalance in the future [10]. Multigene models constructed based on transcriptomics and clinical information can achieve accurate prediction of recurrence risk in hormone receptor-positive breast cancer patients [11]. Thus, it will provide a more accurate reference for the application of postoperative chemotherapy drugs.

With the continuous improvement of hospital information systems and the popularization of digital medical devices, electronic medical record data is growing in huge volume. It provides big data support for the diagnosis and treatment of diseases, but its complexity also brings challenges to data analysis. How can you analyze the electronic medical record data in an intuitive way? The answer lies in its implied knowledge and relationships. Presently, assisting doctors in diagnosis and treatment is one of the important research directions in the field of medical information application.

Electronic medical records are a type of unstructured data. There are numerous models and algorithms in the field of machine learning for this type of data that can effectively analyze patient data [12]. However, due to the multiplicity and high dimensionality of EHR data, it becomes another challenge to present the raw data visually and analyze the results. Visualization techniques combining diverse charts and rich interactions to present data from different levels of abstraction are an effective way to solve these problems.

To this end, this paper uses machine learning models to first analyze electronic medical record data and then present the analysis results through visualization techniques, aiming to help physicians intuitively discover the information implied in inpatient data.

The main contributions of this paper are as follows.

1. Mining similar patient clusters using a dimensional reduction clustering algorithm
2. Using visualization techniques to demonstrate the results of the user-driven analysis to help physicians analyze the correlation of clinical characteristics among different patients
3. Exploring the relationship between different attributes and treatment options based on feature correlation, providing treatment option prediction, assisting preoperative decision making, and improving diagnostic efficiency and treatment effectiveness

The study proceeds by identifying the integrated analysis technology for breast cancer diagnosis and treatment based on combining different data mining techniques combining clinical and genetic data in Section 2. The background studies related to the present study have been highlighted in Section 3. Data collection, analysis, and discussion leading to results proceed to the conclusion of the study at hand.

## 2. Building an Integrated Analysis Technology for Breast Cancer Diagnosis and Treatment Based on Data Mining

This section will explain the building of an integrated analysis technology for breast cancer diagnosis and its treatment based on data mining. The explanation is as follows.

### 2.1. Combining Clinical Data and Genetic Data

Clinically, different diagnosis modules and treatment knowledge can be built through data mining technology by combining clinical data and genetic data of breast cancer to improve the diagnosis and treatment process of breast cancer. Artificial intelligence breast cancer diagnosis and treatment system provide the whole process of disease management for breast cancer patients, including examination, treatment and follow-up, intelligent monitoring, and management of the whole process, optimize the treatment plan in time according to the changes of the disease, improve the treatment effect, and save the treatment cost for patients by enhancing the diagnosis and treatment process [13]. Building different diagnostic and treatment knowledge modules, mainly including accurate clinical diagnosis of breast, surgical treatment, and comprehensive treatment, is helpful in the overall treatment progress of the patient.

### 2.2. Using Data Mining Techniques

Breast cancer artificial intelligence systems use data mining techniques and supercomputer platforms to analyze both diagnostic and therapeutic approaches to breast cancer using genetic testing data. This genetic analysis approach based on big data mining and other genetic screenings for breast cancer and customized precision medicine techniques has been rapidly developing. The Breast Cancer AI System combines medical imaging data with clinical data and provides an accurate diagnosis of breast cancer based on the total amount of data.

Accurate clinical diagnosis includes high-quality, efficient, and standardized clinical examination and a reasonable selection of auxiliary examinations. This includes accurate imaging diagnosis, accurate testing techniques, accurate disease diagnosis (such as different clinical stages), and accurate pathological diagnosis. Precise surgical treatment includes choosing the best time for surgery and selecting the best surgical method. Currently, the most commonly used surgical methods for breast cancer, that is, modified radical surgery and breast-conserving surgery, are available. They must be selected scientifically according to the patient's specific situation and after determining the surgical method. The principles that still need to be selected are the best method, reasonable pathway, and surgical standardization, and determining the perioperative management, including the management of complications, the rational use of antibiotics, the prevention and treatment of surgical complications, and nutritional support are imperative in the procedure [14].

Accurate and comprehensive treatment includes radiotherapy, chemotherapy, endocrine therapy, and molecular targeted therapy. Different irradiation doses are adopted for different conditions of specific patients, etc. For patients with indications for chemotherapy, the dose of chemotherapy and the density and management of adverse effects may be different and should be treated differently. For patients treated with endocrine therapy, menopausal status should be considered in the selection of drugs. Molecular targeted therapy must be clarified with HER2 gene testing results [15]. While informing patients of possible complications, attention should be paid to supportive therapy, treatment of complications, psychotherapy, and rehabilitation training so that patients can obtain the best treatment outcome.

The artificial breast cancer intelligent system will recommend the best treatment plan to the doctor based on the diagnosis. The doctor will expand the relevant treatment tools, according to the stage of the tumor and the patient's physical condition.

### 2.3. Leveraging Clinical Intelligence Decision Support Systems

The emergence of a clinical intelligent decision support system can quickly realize the effective integration of information resources and clinical experience and provide breast cancer surgeons with diagnosis and treatment decisions in complex medical activities, which is manifested as “5 precision.” Precise diagnosis and treatment information is shared in precise information format at the precise time and through precise information channels. The information is shared with the right people at the right time and in the right format. The introduction of a clinical intelligence decision support system in breast cancer treatment can provide doctors with a treatment plan. This plan shall be based on the latest treatment guidelines, research progress, and the most mature clinical experience, which helps breast cancer patients get accurate treatment. In the early screening of breast cancer, the clinical intelligence system gives the location and localization of mass lesions and calcified lesions through the analysis of image data. The computer is used to improve the efficiency of medical film reading, reduce the rate of diagnostic failure and misdiagnosis, and provide quantitative image interpretation reports to help doctors and patients better understand the condition [15].

However, the application of clinical intelligence decision support systems requires attention to the issue of “uncertainty.” This requires breast surgery specialists to make reasonable judgments based on clinical experience and research information. This also indicates that the clinical intelligent decision support system cannot completely replace the role of doctors at present, but it can be an important helper in the precise treatment of tumors such as compensating for the inexperience and knowledge limitations of clinicians. This provides more accurate diagnosis and treatment information, avoiding errors in clinical treatment, ensuring medical quality, and improving medication safety.

## 3. Related Work

Research on visual analytics of medical data has yielded a number of results, and this section presents work related to data mining of electronic medical records and visualization of electronic medical records.

### 3.1. Electronic Medical Record Data Mining

The electronic medical record is a kind of unstructured data, including structured attributes of patients and unstructured textual descriptions, with the characteristics of plurality and high dimensionality. Compared with paper medical records, the electronic medical record has the characteristics of easy storage and convenient query. Diversity refers to more data types; for example, gender belongs to category type data and age belongs to numerical type data. High dimensionality refers to high data dimensions that are used to record multiple attribute values of each patient, such as blood pressure and blood glucose. By mining electronic medical record data, we try to extract structured medical concepts, including disease types, treatment methods, and development patterns. This helps the doctors to develop treatment plans and improve diagnostic efficiency.

Due to the multiplicity and high dimensionality of the data, machine learning or deep learning methods need to be used to extract information from complex electronic medical record data. Paper [16] considered the concept extraction problem as a sequence labeling task and explored various structure learning methods based on RNN feature extraction with the goal of assigning relevant labels to each key entity word in clinical medical records. Word2vec models are used in [17] to transform some clinical concepts in electronic medical records into high-dimensional vectors and then used these vectors to represent patients and used them as the downstream learning task input. A 2-layer neural network is used in [18] to identify osteoporosis and identify the highest risk factors affecting osteoporosis through model reconstruction. An active learning algorithm is proposed in [19] to iteratively identify rare categories in representation data based on user feedback for personalized medicine.

In this paper, cluster features are extracted using clustering and dimensionality reduction algorithms in the data processing phase. SVM models are used to predict treatment options to help physicians analyze the association between attributes and outcomes.

### 3.2. Electronic Medical Record Visualization

The electronic medical record visualization system [20] presents the data of different patients as well as medical behaviors on a timeline. While using it, you can get more information by clicking on the medical events. Inspired by this work, [21] further designed lifelines with line segments to indicate the continuity of medical events and different colors to identify the (normal or abnormal) status of the patient. This helps the physician to have a better grasp of the treatment process and the treatment outcome. To support the visualization of medical events with different temporal granularity and uncertainty, more symbols are used by [22] to represent the temporal information of events more finely, such as minimum duration, and provided additional views to show the temporal relationships of different events. 2-star coordinate plots are used by [23] to show the changes of 12 indicators of patients, with a 1-time interval every 30 min, and different indicators at the same time were plotted with a polygon drawn with connecting lines for different indicators at the same time. The indicators, body organs, and their relationships were visualized with animations and different colors.

Early studies of electronic medical record visualization focused on presenting individual patient records. Compared to textual records, it added graphic coding and simple interaction, and physicians could view patient information intuitively. However, with the development of information technology and the massive accumulation of electronic medical record data, the display of individual patient data alone can no longer meet the needs of physicians. Therefore, the focus on information mining and visual analysis of patient groups has begun to find correlations among patients and search for optimal treatment plans.

Temporal information is an extremely important class of features in electronic medical record data. A large number of studies have analyzed patient time records as sequences of temporal events. Based on Lifelines, Lifelines2, [23] added a comparison function to the time axis display and emphasized the temporal order through alignment, sorting, and filtering operations. This helps the physicians to analyze the trends of medical conditions. Paper [24] designed a comparative visual analysis system for patient groups, using automatic statistical data algorithms to explore the similarities and differences between different patient groups under a user-driven analysis strategy. In addition, work on [10] allows physicians to change medical events in a sequence, such as adding, editing, and deleting, to perform hypothesis analysis to support diagnostic risk prediction. Furthermore, work on event sequence query and recommendation provides technical support for further exploration of EHR data. Unlike temporal event sequence analysis, [17] views EHR data as multimodal data, combining text, image, and audio. The idea of using the similarity of patient records to achieve assisted diagnosis was first proposed by [12], which regarded electronic medical record data as multimodal data. This idea integrated the quantitative analysis of text, image, and audio data into one system. This plan is also the basis for the analysis of similar patient groups in this paper.

## 4. Data and Tasks

The patient's experience in the hospital mainly includes the early screening and examination phase and the treatment phase after the diagnosis is confirmed. Each step of the patient's hospital stay is documented in the electronic medical record, such as admission records, examination results, surgery records and discharge records, etc.

### 4.1. Data

The breast imaging reporting and data system (BI-RADS) classification is the main method of breast cancer assessment and grading, with 0–6 indicating the severity of breast cancer, as shown in Table 1.

Ancillary examinations mainly include the following:

1. Mammography and mammogram include examination of the body position, breast typing, breast impact, lump size, etc. The information that describes the image includes lump size, lump localization, distribution and extent of calcification, etc.
2. Breast ultrasonography mainly contains sonographic descriptions of abnormalities and lesions, such as lesion location, shape, size, surrounding tissues, boundaries, etc. In addition, it also contains the physician's conclusions about the lesion, such as grading and treatment recommendations.
3. Breast MRI contains a comparison of previous medical history and findings, description of imaging findings with breast tissue composition, assessment categories, and management recommendations. It also contains a description of the shape and location of the lesion in question.
4. Immunohistochemistry results are used to assess the infiltration status of breast tissue, determine the type of cancer, help select treatment options, and assess prognosis. The test results include hormone receptor (ER), progesterone receptor (PR), Ki-67 antibodies, CK5/6 antibodies, P63 antibodies, calponin antibodies, CerbB-2 antigen, P120 protein, E-cadherin protein, and other attributes.
5. The pathology report describes the size of the mass, negative and positive lymph nodes, histological grading and type of pathology, surgical plan, etc. The size of the mass was divided into three categories, with boundaries of 2 cm and 4 cm. The pathological histology was divided into grades I to III, and the higher the grading, the higher the malignancy. Negative lymph nodes indicated no metastasis and positive ones indicated metastasis.

### 4.2. Task Description

Physicians and medical researchers want to cascade numerous examination data and find commonalities by analyzing the similarities and differences of various attributes in different patients. They use electronic medical record data to validate the features obtained in clinical practice related to the pathological status and prognosis of breast cancer, such as calculating the correlation or *P*-value of the features to determine the degree of association. At the same time, they want to use machine learning algorithms to automatically analyze relevant data to help in the diagnosis and treatment process, for example, to explore the impact of attributes on treatment options to improve correct decision making.

#### 4.2.1. Details

1. Task 1 (T1) feature correlation analysis: there are correlations between features of the disease, such as simultaneous increase or decrease, and the importance of each feature to the disease varies. Analyzing the relationship between features helps to better understand the disease and its treatment options.
2. Task 2 (T2) construction of different patient clusters: similar patients have similar symptoms and treatment plans, with construction of different patient clusters for all patients in order to analyze the type and characteristics of the disease.
3. Task 3 (T3) analysis and comparison between cohorts: visually comparing and analyzing the similarities and differences of different patient groups, especially the differences in characteristics, helps to better understand the disease course and select treatment options.
4. Task 4 (T4) treatment plan prediction: build machine learning models to predict treatment outcomes based on the patient's current characteristics.
5. Task 5 (T5) demonstrate patient details: present the patient's electronic medical record data and their original treatment reports in order to validate the conclusions.

Based on the above task, this paper designs a system for visual analysis and treatment planning of similar patient groups for breast cancer.

## 5. Visual Analysis of Similar Patient Cohorts

The user's interactive exploration of patient clusters starts with the selection of features. First, the features of interest are selected; then the clustering method and feature reduction algorithm for patient group generation are chosen. Afterward, based on the user selection, the system generates the corresponding results and displays them in the corresponding view. The user explores the relationship between different groups by different methods such as by clicking, boxing, and other interactive methods to view the longitudinal medical history and detailed medical history of individual patients.

### 5.1. Clustered Scatter Plots

The electronic medical record data are of high-dimensional characteristics, so it is necessary to do dimensionality reduction first and then perform clustering to find similar patient groups after being reduced to low-dimensional space. This paper uses scatter plot points to represent patients and different colors to encode the clusters to which the patients belong in order to visualize the dimensionality reduction and clustering results. The coordinates in the scatter plot represent the coordinate values after the high-dimensional features are reduced to two dimensions. Users can gain insight into the degree of clustering among patients in two dimensions through the scatter plot (T2).

In this paper, we choose the multidimensional scaling (MDS) [14–16] algorithm to reduce the high-dimensional attributes of patients to two dimensions. The MDS algorithm calculates the similarity between patients using geometric space (Euclidean space or high-dimensional space) distances. The closer the distance, the more similar the two points.

The distance relationship is kept as monotonic and similar as possible during this process. After dimensionality reduction by MDS, the patients are displayed in two-dimensional spatial coordinates, and clustering algorithms such as K-means are selected for further analysis. The clustering scatter plot will show the clustering process in real time; for example, in Figures 1(a) and 1(b) are the results of selecting K-means algorithm to cluster into two classes and five classes, respectively.

### 5.2. Similar Patient Cohort vs. Cohort Comparison

After selecting the clustering algorithm, the system divides the patients into different groups based on similarity. Each patient is represented by a multidimensional attribute. For Boolean category attributes, the petals are shown if they are owned and hidden if they are not. For numerical attributes and category attributes, the length of the petal is used to represent the petal, and the longer the petal, the greater the value of the patient on the corresponding attribute. Different attributes are displayed in different colors in order to visualize the differences between patients.

After selecting two patient groups, the group comparison histogram will display statistical information on the different attributes to facilitate comparison. The horizontal coordinates show the attributes of the clusters, and for easy differentiation, the 2 adjacent attributes are represented by different background color blocks, the different value intervals of each attribute are counted separately, and the attributes within the same cluster share the same color-coding, and it is the values above and below the horizontal coordinates that need to be compared between the 2 clusters. The vertical coordinate indicates the ratio of the number of patients belonging to the interval to the number of patients in the cluster to which it belongs (*r*), with larger values of *r* indicating more patients in the cluster with attributes in that interval. This design helps to quickly discover the differences between the 2 clusters and uncover patterns of attributes and patient groups of interest. When a physician receives a new patient, he or she can search for the most similar cohort to the patient to obtain the characteristics of that cohort to help develop a treatment plan.

## 6. Visualization of Treatment Plan Design

Based on patient characteristics, prediction models based on breast cancer electronic medical record data can predict treatment plans. It is difficult to make users understand the differences in attributes and characteristics of different patients if only prediction results are provided. To solve this problem, this paper designs a visual analysis system to help doctors analyze the condition and prediction results to assist in developing treatment plans through outlooks and interactions.

### 6.1. Predictive Models

In this paper, we use SVM classification to predict the treatment plan. SVM is a classification model for solving binary classification problems, which is based on the principle of structural risk minimization and finding hyperplane segmentation samples in the sample space.

### 6.2. Matrix Heat Map

Matrix heat maps can be used to represent attribute weights. Since each attribute has a different weight in each classifier, it can be naturally represented by a matrix. Inspired by it, this paper employs a matrix heat map to display the weights of each attribute in each classifier, allowing physicians to quickly identify the most important features.

The system color-codes the feature weights according to their values, as shown in Figure 2. Red indicates positive feature weights, with darker colors indicating larger values; blue indicates negative feature weights, with darker colors indicating the darker the color, the smaller the value. In the matrix heat map, the more prominent the color of the square, the greater influence of the attribute on the classifier, and vice versa. The similarity design of color and background color can remind doctors which attributes have greater influence. At the same time, the upper and lower bounds of the weight intervals displayed in the matrix heat map can be set by the color band on the right side. This enables a filtering operation to hide attributes with too little weight or negative values so that doctors can focus on the intervals of interest.

### 6.3. Classification Chart

To help physicians analyze the classification results of the prediction model, a classification chart was designed. The analysis process requires not only an intuitive understanding of the overall performance of the prediction model but also a detailed analysis of the classification predictions for different patients. The system distinguishes treatment options with different colors to be listed as category aggregation, with each small square indicating a patient and the position of the square indicating the classification result.

Figure 3 shows the prediction results for the category “unilateral mastectomy.” The prediction probability is represented by the left vertical axis, and the “unilateral mastectomy” attribute is used as a vertical axis to divide the prediction sample into two areas, with the right side representing the correct prediction and the left side representing the incorrect prediction. The color of each square is determined by the category to which the patient actually belongs. The color-coding rules are shown in the corresponding legend. The accuracy of the classifier prediction can thus be obtained from the number of squares on the right side, which is the ratio of the number of squares with the same color as the vertical axis to the number of correctly classified samples. In addition, the accuracy of the model can be inspected by the distribution of the squares on the probabilistic prediction vertical axis; that is, the closer the squares to the top, the higher the correct prediction rate. Through these designs, the accuracy and precision of the prediction model can be visualized, and the details of the patient can be obtained by clicking on the squares to complete further investigation.

## 7. Case Study

In this section, different case studies that have been conducted are discussed. The case studies are conducted to help treat the breast cancer patients more effectively. Different case studies are explained above.

### 7.1. General Information

Sixty female patients admitted to our hospital after modified radical surgery after neoadjuvant chemotherapy for breast cancer were selected for the study between August 2018 and August 2019, and the study had been approved by the hospital ethics committee. The patients were divided into a conventional group (*n* = 30 cases) and observation group (*n* = 30 cases) according to the time of starting radiotherapy, in which the mean age of the conventional group was (41.25 ± 8.57) years, and the clinical stage was stage 2 in 18 cases and stage 3 in 12 cases; the mean age of the observation group was (41.32 ± 8.69) years, and the clinical stage was stage 2 in 20 cases and stage 3 in 10 cases. The difference between the two groups at baseline was not statistically significant (*P* > 0.05) and was comparability.

#### 7.1.1. Inclusion Criteria

These criteria include patients who

- Were diagnosed with breast cancer by pathological biopsy
- Underwent neoadjuvant chemotherapy followed by modified radical surgery
- Were of clinical stage 2 to 3

The patients and their families were informed about the study and voluntarily signed the informed consent form.

#### 7.1.2. Exclusion Criteria

These criteria include patients with

- Mental illness or cognitive impairment, unable to communicate normally
- Contraindications to postoperative radiotherapy
- A survival cycle of fewer than 6 months

### 7.2. Results

The total incidence of complications was 36.67% (11/30) in the conventional group and 30% (9/30) in the observation group. When the data of both groups were compared, the difference was not statistically significant (*χ*^2^ = 0.300, *P* > 0.05), as shown in Table 2.

When the data of sixty patients were summarized in the conventional group, the local recurrence rate was 33.33% (10/30) and the progression-free survival was (17.97 ± 4.8) months. The local recurrence rate in the observation group was 16.67% (5/30) and the progression-free survival was (24.01 ± 5.3) months. The difference was statistically significant (*P* < 0.05), as shown in Table 3.

The data of sixty patients were counted, and the scores of patients in the conventional group were (63.54 ± 3.81) for somatic function, (60.85 ± 3.43) for material function, (56.88 ± 2.57) for psychological function, and (61.33 ± 3.52) for a social function. In the observation group, the physical function score was (79.64 ± 2.52), the social function score was (80.04 ± 3.66), and the material function score was (78.73 ± 3.16). The comparison between the two groups showed that the physical function, material function, psychological function, and social function of the patients in the observation group were significantly higher than those in the conventional group (*t* = 19.304 6, 21.438 9, 15.527 6, 22.434 1, *P* < =0.0001, 0.0001, 0.0001, 0.0001).

## 8. Discussion

Breast cancer is a serious threat to women's health and has the second-highest mortality rate after lung cancer. The pathogenesis of this disease is complex and is usually considered to be related to genes, heredity, and diet [25]. Different studies that are conducted at home and abroad have shown that if a patient has an immediate family member with a history of breast cancer, the chance of breast cancer in the family is about two times higher than normal. The most common treatment for breast cancer includes neoadjuvant chemotherapy, which disrupts the mitosis of tumor cells, and chemotherapeutic drugs that bind to DNA after entering the tumor. This helps in preventing tumor cells from synthesizing DNA.

At present, the most effective treatment for breast cancer is mastectomy, but this procedure not only has short efficacy but also causes damage to the breast tissue. On the other hand, modified radical surgery not only achieves tumor eradication but is also less invasive. However, in order to prevent tumor metastasis or recurrence, patients still need adjuvant radiotherapy after modified radical surgery, but the effect of the start time of postoperative radiotherapy on the efficacy of surgery is still unclear [5].

In this study, there was no significant difference in the incidence of radiation pneumonia, radiation dermatitis, hematological toxicity, gastrointestinal reactions, and oral mucosal reactions between patients in the observation group and those in the conventional group. The results suggest that early radiotherapy does not cause further damage to surgically traumatized tissues and can contribute to the early recovery of patients [6]. The result shows that the somatic, physical, and social functions can effectively reflect the important role of early radiotherapy in the improvement of patients' quality of life. This research can help patients relieve postoperative pain to the greatest extent and thus ensure their physical and mental health. The delay of radiotherapy makes the tumor prone to metastasis and recurrence, which is not conducive to the improvement of patients' quality of life, so early radiotherapy after modified radical surgery is recommended [8].

## 9. Conclusions

In conclusion, radiotherapy within 15 weeks after modified radical surgery after neoadjuvant chemotherapy for breast cancer can not only make the local recurrence rate decrease but also prolong the progression-free survival of patients without increasing the complication rate, which greatly helps to improve the quality of life of patients [9]. In this paper, a visual analysis system of breast cancer clusters and treatment plans based on electronic medical records is built to explore the prognostic impact of the start time of radiotherapy after modified radical surgery after neoadjuvant chemotherapy for breast cancer. First, patients with high-dimensional attributes are downscaled and clustered to form patient groups. Then, support vector machine (SVM) models are used to predict treatment plans. Sixty female patients admitted after modified radical surgery after neoadjuvant chemotherapy for breast cancer from August 2018 to August 2019 were selected for the study. Within 15 weeks after neoadjuvant chemotherapy and modified radical mastectomy for breast cancer, radiotherapy not only reduces the local recurrence rate but also prolongs the progression free survival. It does not increase the complication rate, which greatly contributes to the quality of life of patients.

## Figures and Tables

**Figure 1:** Scatter plot of feature dimensionality reduction and clustering process. (a) Real. (b) Predicted.

**Figure 2:** Heat map of the classification weight matrix.

**Figure 3:** Classification chart of prediction results.

**Table 1:** BI-RADS taxonomy.

Classification	Meaning
0	The evaluation is unclear and needs to be assisted
1	No suspicious features
2	Normal, with some benign lesions
3	Highly benign possibility, but follow-up is required
4	Further subdivided into 4a, 4b, and 4C3, the possibility of malignancy is 0∼10%, 10%∼50%, and 50%∼95%, respectively
5	Possibility of high malignancy
6	Biopsy was malignant

**Table 2:** Comparative analysis of patients' complication rates (*n* = 30).

Complication	General group	Observation group
Radiation pneumonia (cases)	0	0
Radiation dermatitis (cases)	1	2
Hematological toxicity (cases)	2	1
Oral mucosal reaction (cases)	6	5
Total complication rate (%)	36.67	30.00

**Table 3:** Comparative analysis of local recurrence rate and progression-free survival of patients (*n* = 30).

Group	Local recurrence rate (%)	Progression-free survival (months, $\bar{x}\pm s$)
General group	33.33	17.97 ± 4.8
Observation group	16.67	24.01 ± 5.3
*x* ^2^/*t* value	7.4015	4.6265
*P* value	0.0065	0.0001

## Data Availability

The datasets used and analyzed during the current study are available from the corresponding author upon reasonable request.
